The article "Exosome-Derived Circ_0094343 Promotes Chemosensitivity of Colorectal Cancer Cells by Regulating Glycolysis via the miR-766-5p/TRIM67 Axis" was published in 2022. Journal: Contrast Media Mol Imaging.

# Exosome-Derived Circ_0094343 Promotes Chemosensitivity of Colorectal Cancer Cells by Regulating Glycolysis via the miR-766-5p/TRIM67 Axis

**DOI:** 10.1155/2022/2878557

**Published:** 2022-07-08

**Authors:** Chen Li, Xu Li

**Affiliations:** ^1^Center for Translational Medicine, The First Affiliated Hospital of Xi'an Jiaotong University, Xi'an, Shanxi 710061, China; ^2^Molecular Testing Center, The First Affiliated Hospital of Jinzhou Medical University, Jinzhou, Liaoning 121011, China; ^3^Key Laboratory for Tumor Precision Medicine of Shaanxi Province, The First Affiliated Hospital of Xi'an Jiaotong University, Xi'an, China; ^4^Key Laboratory of Environment and Genes Related to Diseases (Xi'an Jiaotong University), Ministry of Education of China, Xi'an, China

## Abstract

**Objective:**

Currently, the role of circ_0094343 (circPTEN) on the chemosensitivity of CRC remains to be clarified. This study aimed to investigate the role and mechanism of exosome-delivered circ_0094343 in the proliferation, glycolysis, and chemosensitivity of colorectal cancer (CRC) cells.

**Methods:**

Real-time quantitative polymerase chain reaction (qRT-PCR) was utilized to detect the expression level of circ_0094343, miR-766-5p, and TRIM67 (Tripartite motif-containing 67) in CRC clinical tissue samples and cells, transmission electron microscopy (TEM) to observe the morphology of exosomes, and nanoparticle tracking analysis (NTA) system to measure the diameter of exosomes. Besides, PKH67 fluorescent labeling was applied for assessing the level of exosome uptake by cells, MTT and cell clone formation assays for detecting cell proliferation and clone formation, respectively, and related kits for checking the glucose consumption, lactate production, and extracellular acidification rate (ECAR) in cells. Dual-luciferase reporter (DLR) gene assay was used for verifying the targeting relationship between circ_0094343 and miR-766-5p, miR-766-5p and TRIM67, RNA immunoprecipitation (RIP) experiment for the interaction between circ_0094343 and miR-766-5p, and Western blot for the protein level of exosome surface antigens (HSP70, CD63) and TRIM67 in cells in exosomes and cell lysates.

**Results:**

circ_0094343 was significantly downregulated in CRC tissues, chemotherapy-resistant CRC tissues, and metastatic CRC tissues. Moreover, exosomes-carried circ_0094343 played an inhibitory role in the proliferation, clone formation and glycolysis of HCT116 cells. Meanwhile, it could also improve the chemosensitivity of HCT116 cells to 5-fluorouracil (5-FU), oxaliplatin (L-OHP), and doxorubicin (Dox). Additionally, circ_0094343 acted as a sponge for miR-766-5p, and miR-766-5p targeted and regulated TRIM67. In CRC tissues, miR-766-5p expression was negatively correlated with TRIM67 expression, while circ_0094343 was positively associated with TRIM67. Further, mechanistic validation also demonstrated that circ_0094343 could inhibit HCT116 cell proliferation, clone formation, glycolysis, and chemotherapy resistance via the miR-766-5p/TRIM67 axis.

The article "Exosome-Derived Circ_0094343 Promotes Chemosensitivity of Colorectal Cancer Cells by Regulating Glycolysis via the miR-766-5p/TRIM67 Axis" was published in 2022. Journal: Contrast Media Mol Imaging.

**Conclusion:**

circ_0094343 inhibited the proliferation, clone formation and glycolysis of CRC cells and improved their chemosensitivity to various chemotherapeutic drugs via the miR-766-5p/TRIM67 axis. This finding may provide new insights into the treatment of CRC.

## 1. Introduction

As one of the most common malignant tumors in the world, colorectal cancer (CRC) represents the second and third most incident cancer in males and females, accounting for the third and fourth leading cancer-related deaths, respectively [1]. In fact, only 5% to 10% of CRC belongs to familial hereditary diseases caused by familial adenomatous polyposis (FAP), and more than 90% of CRC belongs to sporadic tumors [2]. The recognition of the occurrence, development, and treatment of CRC have been greatly enhanced due to modern medical level improvement [3, 4]. Nevertheless, the specific indicators for the early diagnosis of CRC are still insufficient because most patients have already entered the middle and late stages by the time they are diagnosed [3, 4]. Moreover, the 5-year survival rate is less than 10% in advanced patients with invasive and metastatic CRC [3, 4]. Additionally, about 60% of advanced patients with metastatic CRC would suffer liver metastases [5]. In recent years, despite remarkable breakthroughs in therapeutic modalities such as chemotherapy and targeted therapy, drug resistance is still the main obstacle for successful treatment in CRC. Therefore, it is an urgent and important clinical requirement to seek suitable markers for CRC screening and early diagnosis and methods for improving CRC chemosensitivity.

Exosomes, as nanoscale (30–100 nm) extracellular vesicles, can be secreted by most types of cells and circulated in body fluids (blood, urine, saliva, and breast milk) [6]. Studies have disclosed that exosomes can encapsulate multiple contents (various growth factors, proteins, lipids, nucleic acids, circular RNAs (circRNAs), miRNAs) and transport them to target cells to play an important role [7]. In recent years, many studies have revealed that exosomes exert significant functions in the malignant behavior of CRC. For example, Lan et al. found that miRNA-containing exosomes derived from M2 macrophages could promote cell migration and invasion of colon cancer [8]. Hu et al. indicated the high correlation of the highly expressed exosome miR-92a-3p with the metastasis and chemotherapy resistance in CRC patients [9]. All in all, the above suggested that exosomes may play a role in the malignant behavior of CRC through their contents.

The article "Exosome-Derived Circ_0094343 Promotes Chemosensitivity of Colorectal Cancer Cells by Regulating Glycolysis via the miR-766-5p/TRIM67 Axis" was published in 2022. Journal: Contrast Media Mol Imaging.

CircRNA is a new type of endogenous RNA with a covalent closed-loop structure [10]. CircRNAs can not only bind to miRNAs or proteins to exert various functions but can also be sorted into extracellular vesicles together with other nucleic acids, lipids, and proteins [11]. When exosomes are secreted from cells into body fluids, circRNAs, as one of the contents of exosomes, initiate their circulation through body fluids and activate biological functions. Presently, several studies have stated that circRNAs can act as miRNA molecular sponges to participate in the pathophysiological processes of CRC cells such as proliferation, migration, invasion, and apoptosis, and circRNAs are rated to the radiosensitivity of CRC [12–14]. Besides, circ_0055625 can activate the ITGB8 signaling pathway via sponging miR-106b-5p, thereby promoting the progression of CRC [15]. Thus, the circRNA/miRNA/target gene/target protein axis may be important in CRC.

It has been reported that exosome-carried circRNAs play an important role in the malignant behavior of CRC. For example, Zhao et al. claimed that exosome-delivered circ_0000338-enhanced CRC resistance to 5-fluorouracil (5-FU) through the negative regulation of miR-217 and miR-485-3p [16]. Zhao et al. showed that exosomes from CD133 cells with circ-ABCC1 could regulate stemness, spheroidization, and metastasis of CRC cells [17]. The above suggested the great potential of exosomes that encapsulated circRNAs in CRC. This study aimed to provide a meaningful experimental basis for searching biomarkers of CRC and resolving chemoresistance in CRC by investigating the effect and mechanism of exosome-delivered circ_0094343 on the proliferation, glycolysis, and chemoresistance of CRC cells.

## 2. Materials and Methods

### 2.1. Clinical Samples

Twenty cases of tumor tissues (CRC) and twenty cases of histologically normal para-carcinoma tissues (adjacent tissue) were collected from CRC patients who underwent surgery in the First Affiliated Hospital of Xi'an Jiaotong University. According to whether the tumor is sensitive to 5-FU, the tumor tissues were divided into sensitive group and resistance group. According to whether the tumor has metastasis, the tumor tissues were divided into metastasis group and nonmetastasis group. Besides, this study was approved by the Ethics Committee of the First Affiliated Hospital of Xi'an Jiaotong University (KYLL202016), and all experimental steps were carried out following the approved guidelines. All patients volunteered to be involved in the collection of clinical tissues and signed informed consent.

The article "Exosome-Derived Circ_0094343 Promotes Chemosensitivity of Colorectal Cancer Cells by Regulating Glycolysis via the miR-766-5p/TRIM67 Axis" was published in 2022. Journal: Contrast Media Mol Imaging.

### 2.2. Cell Culture and Transfection

Human normal colon epithelial cells NCM460 and CRC cells HCT116 were purchased from the National Collection of Authenticated Cell Cultures. Then, HCT116 and NCM460 cells were cultured in Dulbecco's Modified Eagle Medium (DMEM) and Roswell Park Memorial Institute Medium (RPMI)-1640 (Gibco, USA) containing 10% fetal bovine serum (FBS, Gibco, USA) and 1% penicillin-streptomycin (Gibco, USA), respectively. All cells were cultured in an incubator at 37°C with 5% CO_2_ and 95% humidity.

Negative vector and overexpression vector pcDNA3.1 circ_0094343 (circ), as well as negative mimics and overexpression miR-766-5p mimics, were purchased from Guangzhou Ribobio Biotechnology Co., Ltd. NCM460 and HCT116 cells in logarithmic growth phase were collected and seeded in 6-well plates. The transfection was performed when the cell confluence reached about 80%. Specifically, the negative vector and overexpression vector pcDNA3.1 circ_0094343 (circ) were transfected into NCM460 cells, respectively. Afterward, exosomes were extracted and named exo-vector and exo-circ accordingly. In this study, HCT116 culture and transfection grouping were as follows: (1) In the NC group, HCT116 cells were cocultured with phosphate-buffered saline (PBS) solution; in the exo-vector group, HCT116 cells were cocultured with exo-vector; in the exo-circ group, HCT116 cells were cocultured with exo-circ; (2) in the mimics NC group, negative mimics were transfected into HCT116 cells; in the miR-766-5p mimics group, miR-766-5p mimics were transfected into HCT116 cells; (3) in the NC group, HCT116 cells were cocultured with PBS solution; in the exo-circ group, HCT116 cells were cocultured with exo-circ; in the miR-766-5p mimics group, miR-766-5p mimics were transfected into HCT116 cells; in the exo-circ + miR-766-5p mimics group, HCT116 cells transfected with miR-766-5p mimics were cocultured with exo-circ. All above transfections were carried out following the instructions of Lipofectamine 2000 (Invitrogen, USA). After 48 h, the cells were collected.

### 2.3. Exosome Isolation

*Labeling and Identification.* Exosomes were extracted from the cell culture supernatant and suspended in PBS according to the instructions of the Exo Quick-TC kit (Shanghai Lan Shan Biological Technology, China). Then, transmission electron microscopy (TEM) was utilized to identify exosome morphology. Besides, bicinchoninic acid (BCA) protein assay (Solarbio, China) was applied for the measurement of the protein content; Western blot for the detection of the expression of exosome-specific markers CD63 and HSP70; and Nanoparticle Tracker (NTA) system for determination of the size of vesicles [18].

The article "Exosome-Derived Circ_0094343 Promotes Chemosensitivity of Colorectal Cancer Cells by Regulating Glycolysis via the miR-766-5p/TRIM67 Axis" was published in 2022. Journal: Contrast Media Mol Imaging.

Based on the published protocol by Bang et al., the exosomes were fluorescently labeled according to the instructions of the PKH67 fluorescent cell kit (Sigma, USA) [19]. After the PKH67-labeled exosomes were diluted with PBS, 1 h ultracentrifugation at 150000 g was performed at 4°C to remove unincorporated dye contamination in the exosome labeling reaction. Next, purified PKH67 exosomes were cocultured with HCT116 cells for 48 h, and the cells were fixed with 4% paraformaldehyde (Beyotime, China). Besides, the cells were stained with DAPI (Beyotime, China), and then the nucleus could be observed. Finally, the distribution of cells and exosomes were observed under a fluorescence microscope.

### 2.4. Real-Time Quantitative Polymerase Chain Reaction (qRT-PCR)

The total RNA was extracted from the collected cells or tissues using Trizol reagent (Solarbio, China). Before extraction, the tissues were first homogenized in a tissue homogenizer. Then, Nanodrop was used to determine the concentration and purity of the extracted RNA. Furthermore, cDNA was synthesized via reverse transcription following the instructions of the PCR kit (Takara, Japan). Then, cDNA was utilized to determine the relative expression level of circ_0094343, miR-766-5p, and TRIM67 (Tripartite motif-containing 67) following the instructions of the real-time PCR kit (Takara, Japan). U6 and GAPDH served as internal controls, and data analysis was performed using the 2^−ΔΔCt^ method. The primer sequences used are shown in Table 1 [20].

### 2.5. MTT Assay

Transfected cells were collected, and the concentration was adjusted to 5 × 10^4^ cells/ml. Then, 100 *μ*L of cell suspension was seeded in a 96-well plate and cultured in a cell incubator. After cell adhesion, the culture was discontinued. Subsequently, the exosomes (exo-vector or exo-circ) extracted from NCM460 cells were added into cell suspension, and the cell proliferation ability was measured at 0 h and 24 h after cell adhesion according to the instructions of the MTT kit, respectively. Afterward, 10 *μ*L of MTT solution (5 mg/ml) was added to each well for another 4 h culture. Then, 100 *μ*L of Formazan dissolving solution was supplemented to each well for continual 3-4 h incubation. After the purple crystals were completely dissolved, the absorbance at 570 nm was measured using a microplate reader. At least six replicate wells were set for each group. In the chemosensitivity detection experiment of cells, exosomes and different concentrations (0 M, 0.1 M, 0.5 M, 1 M, 5 M, 10 M) of chemotherapeutic drugs (5-FU, oxalicylic platinum (L-OHP), and doxorubicin (Dox)) were required to be added at the same time. Other steps were the same as those in the proliferation experiment.

The article "Exosome-Derived Circ_0094343 Promotes Chemosensitivity of Colorectal Cancer Cells by Regulating Glycolysis via the miR-766-5p/TRIM67 Axis" was published in 2022. Journal: Contrast Media Mol Imaging.

### 2.6. Cell Clone Formation Assay

Cells in the logarithmic growth phase were collected and pipetted into a single cell suspension. Later, the cell suspension was seeded into a 12-well plate at 400 cells/well, followed by static culture at 37°C with 5% CO_2_ for 2-3 weeks. After rinsing with PBS, the cells were fixed with 4% paraformaldehyde (Beyotime, China) for 15 min, and crystal violet solution (Beyotime, China) was adopted for another 15 min staining. Finally, the number of clones was counted under a microscope.

### 2.7. Detection of Glucose Consumption, Lactate Production, and Extracellular Acidification Rate (ECAR)

The level of glucose consumption, lactate production, and ECAR were measured according to the instructions of the glucose detection kit, lactate detection kit, and ECAR kit, respectively. Specifically, the cell culture medium supernatant was collected and diluted after 48 h transfection. Subsequently, the diluted solution was added to a 96-well plate. Besides, the standard wells were set up, and the working solution was added. A 20-minute reaction was performed at 37°C, and then the optical density (OD) of each well was determined at a wavelength of 570 nm. A standard curve was drawn to calculate glucose content, lactate content and ECAR [21].

### 2.8. Dual-Luciferase Reporter (DLR) Assay

Transfection was performed when the confluence of 293T cells reached 80%–90%. The constructed circ_0094343 or TRIM67 wild-type WT and mutant MUT dual-luciferase reporter vectors and miR-776-5p mimics or mimics NC were cotransfected into cells, respectively. After transfection, another 48 h culture was conducted. Then the cells were collected and lysed at ambient temperature for 20 min. After centrifugation, the supernatant was collected. Next, luciferase substrate was added to the supernatant, and the luciferase activity was detected using a luminometer. Besides, the renilla luciferase enzyme activity served as the internal control to calculate the relative firefly luciferase activity [22].

### 2.9. RNA Immunoprecipitation (RIP) Experiment

The binding of circ_0094343 and miR-766-5p to AGO2 protein was determined according to the EZ-Magna RIP RNA-Binding Protein Immunoprecipitation Kit instructions (Millipore, USA). Specifically, the cells were lysed with an equal volume of RIP lysis buffer on ice for 5 min. Then, the cell lysates were incubated with magnetic beads conjugated with Ago2 or IgG antibodies (Abcam, UK). Finally, qRT-PCR was utilized to measure the enrichment of circ_0094343 and miR-766-5p.

The article "Exosome-Derived Circ_0094343 Promotes Chemosensitivity of Colorectal Cancer Cells by Regulating Glycolysis via the miR-766-5p/TRIM67 Axis" was published in 2022. Journal: Contrast Media Mol Imaging.

### 2.10. Western Blot

Cells, exosomes, and cell lysates were lysed on ice with RIPA lysis buffer (Solarbio, China). After the total protein was extracted, sonication was performed in an ice bath, and centrifugation was conducted at 10,000 rpm at 4°C for 20 min. Then, the protein supernatant was collected. A BCA kit (Solarbio, China) was used to check the protein concentration. Further, 20 *μ*g of total protein was separated by sodium dodecyl sulfate-polyacrylamide gel electrophoresis (SDS-PAGE) and transferred to polyvinylidene fluoride (PVDF) membranes. After blocking with 5% nonfat milk blocking solution at ambient temperature for 1–2 h, diluted primary antibodies (anti-HSP70, anti-CD63, anti-TRIM67, and anti-*β*-actin, CST, USA) were added for incubation overnight at 4°C. After washing the membranes twice with phosphate-buffered saline with tween (PBST), a diluted enzyme-labeled secondary antibody (Zhongshan Golden Bridge, China) was added for another 1-h incubation at ambient temperature. After washing with PBST for another three times, electrochemiluminescence (ECL) luminescent solution was added (Beyotime, China) for following exposure and photography in a gel imager. Image-pro plus software was used to analyze the gray value of the protein bands, and *β*-actin served as an internal control for the analysis of the relative expression level of the target protein.

### 2.11. Statistical Analysis

The results were expressed as mean ± standard deviation (SD) and plotted using GraphPad Prism 9 software. SPSS 24.0 and Graphpad prism 9 software were used for statistical analysis. The *t*-test was used for comparison between two groups and one-way analysis of variance for comparison between multiple groups. *P* <0.05 was regarded as the criterion for statistically significant differences. All experiments were repeated at least 3 times.

## 3. Results

### 3.1. Downregulation of Circ_0094343 Expression in Colorectal Cancer Tissues

To clarify the relation of circ_0094343 with the occurrence, metastasis and chemotherapy resistance of CRC, circ_0094343 expression level in clinical tissues was examined. As a result, the circ_0094343 expression level in the CRC group was much lower than in the adjacent tissue group (*P* < 0.01). Compared with the sensitive group, the resistance group exhibited a remarkably decreased circ_0094343 expression level (*P* < 0.01). However, compared with the nonmetastasis group, the metastasis tissue showed an obvious reduction in circ_0094343 expression level (*P* < 0.01). The above suggested that circ_0094343 may be related to the occurrence, metastasis, and chemotherapy resistance of CRC (Figures 1(a)–1(c)).

The article "Exosome-Derived Circ_0094343 Promotes Chemosensitivity of Colorectal Cancer Cells by Regulating Glycolysis via the miR-766-5p/TRIM67 Axis" was published in 2022. Journal: Contrast Media Mol Imaging.

### 3.2. Characterization of NCM460 Cell Exosomes

Subsequently, to further explore the effect of exosome-derived circ_0094343 on CRC cells, we extracted exosomes from NCM460 cells for the following identification. After negative staining of exosomes with uranyl acetate, the findings revealed round or oval vesicles with a membrane-like structure in the exo-vector group and exo-circ group under a transmission electron microscope (Figure 2(a)). Besides, the NTA assay showed that the average diameter of exosomes was about 136 nm in the exo-vector and exo-circ groups, and the particle size ranged from 75 to 150 nm (Figure 2(b)). In addition, compared with the cell lysate group, the protein levels of exosome markers HSP70 and CD63 in exosomes were significantly increased in the exo-vector and exo-circ groups. The above findings indicated successful extraction of exosomes from the cells (Figure 2(c)).

The level of circ_0094343 in the extracted exosomes was determined, and the outcomes disclosed that the circ_0094343 expression level in exosomes in the exo-circ group was far higher than that in the exo-vector group (*P* < 0.01) (Figure 2(d)). To explore the interaction between the extracted exosomes and HCT116, we labeled exosomes with PKH67 and observed their distribution in HCT116. According to the results of immunofluorescence detection, the PKH67 fluorescence signal could be observed in HCT116 cells in the exo-vector and exo-circ groups. However, there was no PKH67 signal in the NC group. The above findings suggested that HCT116 cells possibly played a role in absorbing exosomes through endocytosis (Figure 2(e)).

### 3.3. Exosome-Derived Circ_0094343 Inhibits the Proliferation and Glycolysis of HCT116 Cells

Further, the effects of exosome-derived circ_0094343 on the proliferation and glycolysis of HCT116 cells were determined. Compared with the exo-vector group, the exo-circ group presented a remarkable decrease in the proliferation rate, clone formation, glucose consumption, lactate production, and ECAR in HCT116 cells (*P* < 0.05). Nevertheless, the above indicators were not observed obvious differences between the NC group and the exo-vector group (Figures 3(a)–3(f)). Briefly, it could be concluded that exosome-derived circ_0094343 could inhibit the proliferation and glycolysis of HCT116 cells.

### 3.4. Exosome-Derived Circ_0094343 Enhances the Chemosensitivity of HCT116 Cells

Furthermore, we explored the correlation of exosome-derived circ_0094343 with the chemotherapy resistance of HCT116. The outcomes are shown in Figures 4(a)–4(c). Specifically, the survival rate of HCT116 cells in the exo-circ group was significantly lower than that in the exo-vector group under the treatment of 5-FU, L-OHP, and Dox (*P* < 0.01). However, the chemosensitivity of HCT116 cells to 5-FU, L-OHP, and Dox was not significantly different between the NC and the exo-vector groups. The above indicated that exosome-derived circ_0094343 enhanced the chemosensitivity of HCT116 cells to 5-FU, L-OHP, and Dox.

The article "Exosome-Derived Circ_0094343 Promotes Chemosensitivity of Colorectal Cancer Cells by Regulating Glycolysis via the miR-766-5p/TRIM67 Axis" was published in 2022. Journal: Contrast Media Mol Imaging.

### 3.5. Circ_0094343 Acts as a Sponge for miR-766-5p

To further investigate whether circ_0094343 exerts its function by binding to miRNAs, the CircRNABase website was used to predict the target miRNAs of circ_0094343. The prediction results revealed that circ_0094343 could target and bind to miR-766-5p (Figure 5(a)). Then, the DLR gene assay was performed to verify the targeting relationship between circ_0094343 and miR-766-5p. The findings suggested that cotransfection of miR-766-5p mimics markedly inhibited the luciferase activity of circ_0094343-WT but not the activity of circ_0094343-MUT vector (Figure 5(b)). Besides, RIP experiment results disclosed that, compared with the IgG group, the recruitment level of circ_0094343 and miR-766-5p in the AGO2 group was remarkably increased (Figures 5(c) and 5(d)). All in all, the targeting relationship was confirmed between circ_0094343 and miR-766-5p. Additionally, we detected the expression level in clinical samples and cells. We found significantly higher miR-766-5p expression levels in tissues of the CRC group than in the adjacent tissue group (*P* < 0.01, Figure 5(e)). Moreover, a negative correlation was shown in the expression level of miR-766-5p and circ_0094343 in CRC tissues (Figure 5(f)). In addition, the miR-766-5p expression level in HTC116 cells in the exo-circ group was significantly lower than in the exo-vector group (*P* < 0.01, Figure 5(g)). These findings thereby suggest that circ_0094343 acts as a sponge for miR-766-5p.

### 3.6. miR-766-5p Targets TRIM67

Based on the TargetScan online database, miR-766-5p was further discovered as able to target and regulate TRIM67, and the target sequences are shown in Figure 6(a). According to the outcomes of the DLR assay, transfection of miR-766-5p mimics could significantly inhibit the luciferase activity of cells in the TRIM67-WT group (*P* < 0.01), while the luciferase activity of the cells in the TRIM67-MUT group was not significantly affected (Figure 6(b)). The above findings indicated that miR-766-5p could target TRIM67. Further expression detection revealed that compared with the adjacent tissue, the TRIM67 expression level in the CRC tissue was significantly reduced (*P* < 0.01, Figure 6(c)). Moreover, TRIM67 expression was positively correlated with circ_0094343 expression in the CRC tissue (Figure 6(d)) while negatively correlated with miR-766-5p expression (Figure 6(e)). Furthermore, the protein and mRNA expression level of TRIM67 was significantly decreased after miR-766-5p mimics overexpressed miR-766-5p in HCT116 cells (*P* < 0.01, Figures 6(f)–6(h)). In addition, an obvious upregulation was observed in the expression level of TRIM67 in cells of the exo-circ group compared with the exo-vector group (*P* < 0.01, Figure 6(i)). All results above suggested that miR-766-5p could target and regulate TRIM67.

The article "Exosome-Derived Circ_0094343 Promotes Chemosensitivity of Colorectal Cancer Cells by Regulating Glycolysis via the miR-766-5p/TRIM67 Axis" was published in 2022. Journal: Contrast Media Mol Imaging.

### 3.7. Exosome-Derived Circ_0094343 Inhibits the Proliferation and Glycolysis and Improves the Chemosensitivity of HCT116 Cells via the miR-766-5p/TRIM67 Axis

It remains unclear whether exosome-derived circ_0094343 inhibited CRC cell proliferation, glycolysis, and chemotherapy resistance through the miR-766-5p/TRIM67 axis. To further investigate this question, CRC cells were simultaneously treated with exo-circ_0094343 (exo-circ) and miR-766-5p mimics. Then, an evaluation was performed on the proliferation, glycolysis, and chemotherapy resistance of the cells (Figures 7(a)–7(l)). In comparison with the cells in the NC group, TRIM67 expression was significantly increased in the exo-circ group but remarkably decreased in the miR-766-5p mimics group. Besides, TRIM67 expression in the cells of the exo-circ + miR-766-5p mimics group was significantly lower than the exo-circ group while significantly higher than that of the miR-766-5p mimics group (Figures 7(a)–7(c)).

On the one hand, compared with the NC group, a significant decrease was presented in the proliferation rate, clone formation number, glucose consumption, lactate production, and ECAR level of cells in the exo-circ group (*P* < 0.01), while the above indicators were significantly increased in cells of the miR-766-5p mimics group (*P* < 0.01). On the other hand, the proliferation rate, clone formation, glucose consumption, lactate production, and ECAR level of the exo-circ + miR-766-5p mimics group were significantly higher than those in the exo-circ group (*P* < 0.05) but far lower than those in the miR-766-5p mimics group (*P* < 0.01) (Figures 7(d)–7(i)). In addition, despite the significant decrease in the exo-circ group, the chemotherapy resistance of cells to 5-FU, L-OHP, and Dox was significantly increased in the miR-766-5p mimics group. The survival rate of cells in the exo-circ + miR-766-5p mimics group was remarkably higher than the exo-circ group while significantly lower than the miR-766-5p mimics group (Figures 7(j)–7(l)). The above findings indicated that exosome-derived circ_0094343 inhibited the proliferation and glycolysis of HCT116 cells and improved chemosensitivity to various chemotherapeutic drugs via the miR-766-5p/TRIM67 axis.

The article "Exosome-Derived Circ_0094343 Promotes Chemosensitivity of Colorectal Cancer Cells by Regulating Glycolysis via the miR-766-5p/TRIM67 Axis" was published in 2022. Journal: Contrast Media Mol Imaging.

## 4. Discussion

Related studies showed that circRNAs are stably enriched in exosomes and can be detected in circulating blood and urine [23]. Accumulating evidence has revealed that exosomal circRNAs play a key role in tumor growth [7], immune escape [7], angiogenesis [24], metastasis [25], and drug resistance formation [26] in CRC. Specifically, exosomes can not only be incorporated by many types of cells, including macrophages, but also serve as intercellular messengers—they can transfer circRNAs for cells. Moreover, exosomal circRNAs are considered to have higher sensitivity and specificity than individual carcinoembryonic antigens and carbohydrate antigens [27]. In this study, circ_0094343 was downregulated in CRC tissues, chemotherapy-resistant CRC tissues, and metastatic CRC tissues. Furthermore, exosome-delivered circ_0094343 could inhibit the proliferation, clone formation, and glycolysis and improve the chemosensitivity of HCT116 cells. Li [28] also revealed significantly low circ_0094343 expression in CRC tissues. Besides, they reported that the upregulation of circ_0094343 could inhibit the proliferation, clone formation, migration, and invasion while promoting apoptosis of CRC cells [28]. All in all, circ_0094343 may exert an anticancer effect on cancer.

Researches have shown that miR-766-5p expression in CRC tissues is significantly higher than in normal tissues [29]. Moreover, downregulated miR-766-5p expression can inhibit the proliferation, migration, and invasion, and promote the apoptosis of cancer cells [29]. Similar to the previous findings, this study observed an obvious elevation of the expression level of miR-766-5p in CRC tissues. TRIM67 is a protein-coding gene with 84 kDa in length [30]. As a member of the TRIM protein family, TRIM67 locates on the long arm of chromosome 1 and contains a RING domain, one or two B-box domains, a coiled-coil domain (coiled-coil), and a C-terminal structure [30]. Multiple studies have indicated that TRIM protein family members are involved in various biological processes such as cell proliferation, differentiation, development, anti-HIV, carcinogenesis, and apoptosis [31]. In this study, TRIM67 was significantly underexpressed in CRC. The study by Wang et al. also showed that TRIM67 could inhibit the occurrence and progression of CRC by activating p53 [32]. Additionally, Liu et al. disclosed the remarkably downregulated TRIM67 expression in CRC tissues, and TRIM67 expression was related to clinical stage, invasion, tumor size, lymph node metastasis, and staging; besides, TRIM67 played an inhibitory role in the proliferation, migration and invasion of CRC cells by mediating MAPK11 [33]. All of the above findings suggested that TRIM67 may exert an anticancer effect on CRC.

The article "Exosome-Derived Circ_0094343 Promotes Chemosensitivity of Colorectal Cancer Cells by Regulating Glycolysis via the miR-766-5p/TRIM67 Axis" was published in 2022. Journal: Contrast Media Mol Imaging.

In this study, *in vitro* experiments demonstrated that exosome-derived circ_0094343 inhibited the glycolysis, proliferation and clone formation of CRC cells via the miR-766-5p/TRIM67 axis and, at the same time, enhanced the sensitivity to various chemotherapeutic drugs (5-FU, L-OHP, and Dox). Exosome-derived circ_0094343 is of considerable value as a diagnostic marker for chemotherapy-resistant CRC patients. It provides a promising therapeutic intervention for overcoming 5-FU, L-OHP, and Dox resistance in CRC patients. However, uncertainty still remains in the role of exosome-derived circ_0094343 *in vivo*. Therefore, more *in vivo* experiments must be performed for further verification.

## 5. Conclusion

In conclusion, as well as improving the chemosensitivity to various chemotherapeutic drugs, exosome-delivered circ_0094343 inhibits the proliferation, clone formation, and glycolysis of CRC cells (HCT116) by regulating the miR-766-5p/TRIM67 axis. Moreover, this study offers a new research perspective for exploring CRC progression and chemotherapy resistance, which is of great significance in the diagnosis and chemotherapy sensitization of CRC.

## Figures and Tables

**Figure 1:** Downregulation of circ_0094343 expression in the tissues of colorectal cancer patients. (a)–(c), qRT-PCR for detecting circ_0094343 expression level in colorectal cancer (CRC) tissues and corresponding para-cancerous tissues (a), chemotherapy-sensitive and chemotherapy-resistant CRC tissues (b), as well as metastatic and nonmetastatic CRC tissues (c). ^*∗∗*^*P* < 0.01.

**Figure 2:** Characterization of exosomes from NCM460 cells. (a) After negative staining of exosomes with uranyl acetate, the morphology of exosomes in the exo-vector group and the exo-circ group was observed by transmission electron microscopy (TEM); (b) nanoparticle tracker to detect the diameter of exosomes in the exo-vector group and the exo-circ group; (c) Western blot to determine the protein expression level of HSP70 and CD63 in exosomes and cell lysates in each group; (d) qRT-PCR for determination of circ_0094343 expression level in exosomes in each group; (e) PKH67 fluorescent labeling was performed to determine the level of exosome uptake by HCT116 cells. ^*∗∗*^*P* < 0.01.

**Figure 3:** Exosome-derived circ_0094343 inhibits the proliferation and glycolysis of HCT116 cells. (a) MTT assay to detect the effect of exosomes on the proliferation rate of HCT116 cells in each group. (b), (c) The role of exosomes in the clone formation of HCT116 cells was measured in each group using clone formation assay. (d)–(f) Related kits to test the effect of exosomes of each group on glucose consumption (d), lactate production (e), and ECAR (f) in HCT116 cells. ^*∗∗*^*P* < 0.01 and ^*∗*^*P* < 0.05.

The article "Exosome-Derived Circ_0094343 Promotes Chemosensitivity of Colorectal Cancer Cells by Regulating Glycolysis via the miR-766-5p/TRIM67 Axis" was published in 2022. Journal: Contrast Media Mol Imaging.

**Figure 4:** Exosome-derived circ_0094343 enhances the chemosensitivity of HCT116 cells to various chemotherapeutic drugs. (a)–(c) MTT for detection of the survival rate of HCT116 cells in each group under different concentrations of 5-FU (a), L-OHP (b), and dox (c) treatment. ^*∗∗*^*P* < 0.01 vs. exo-vector.

**Figure 5:** Circ_0094343 acts as a sponge for miR-766-5p. (a) CircRNABase website to predict the targeting sequences of circ_0094343 and miR-766-5p; (b) DLR gene assay to verify the targeting relationship between circ_0094343 and miR-766-5p; (c), (d) RIP experiments for verification of the direct binding of circ_0094343 and miR-766-5p; (e) qRT-PCR for detecting the expression level of miR-766-5p in tissues of the CRC group and adjacent group; (f) Pearson correlation for the analysis of the relationship between circ_0094343 and miR-766-5p expression in CRC tissues; (g) qRT-PCR to measure miR-766-5p expression level in the NC group, exo-vector group and exo-circ group. ^*∗∗*^*P* < 0.01.

**Figure 6:** miR-766-5p targets TRIM67. (a) TargetScan website predicted the targeting sequences of miR-766-5p and TRIM67; (b) DLR gene assay verified the targeting relationship between circ_0094343 and miR-766-5p; (c) qRT-PCR measured TRIM67 expression level in the CRC tissue and adjacent tissue; (d), (e) Pearson correlation analysis analyzed the correlation between miR-766-5p and TRIM67 expression in CRC tissue (d) as well as the association between circ_0094343 and TRIM67 expression (e); (f) qRT-PCR determined the expression level of miR-766-5p and TRIM67 in HCT116 cells after miR-766-5p mimics and mimicked NC treatment; (g), (h) Western blot for detection of the protein expression level of TRIM67 in HCT116 cells after miR-766-5p mimics and mimics NC treatment; (i) qRT-PCR detected the expression level of TRIM67 in cells of each group. ^*∗∗*^*P* < 0.01.

**Figure 7:** Exosome circ_0094343 inhibits the proliferation and glycolysis and improves the chemosensitivity of HCT116 cells through the miR-766-5p/TRIM67 axis. (a) qRT-PCR for detection of the mRNA expression level of TRIM67 in cells of each group; (b), (c) Western blot was used to determine the protein expression level of TRIM67 in cells of each group; (d) MTT for checking the proliferation rate of cells in each group; (e), (f) The clone formation ability of the cells in each group was evaluated using clone formation assay; (f)–(i), kits to detect the glucose consumption level (g), the lactate production level (h), and the level of ECAR (i) of the cells in each group; (j), (l) MTT for determination of the survival rate in each group of cells treated with different concentrations (0, 0.5, 1, 5, 10, 50 *μ*M) of 5-FU (j), L-OHP (k), and Dox (l). ^*∗∗*^*P* < 0.01 vs., NC, ^##^*P* < 0.01 and ^#^*P* < 0.05 vs., exo-circ, ^&&^*P* < 0.01 vs., miR-776-5p mimics.

The article "Exosome-Derived Circ_0094343 Promotes Chemosensitivity of Colorectal Cancer Cells by Regulating Glycolysis via the miR-766-5p/TRIM67 Axis" was published in 2022. Journal: Contrast Media Mol Imaging.

**Table 1:** qRT-PCR primer sequences.

Gene name	Primer sequences (5′ to 3′)
circ_0094343	F AAAAAGCAATGAGCCATAGAAA
	R ACGCCTTCAAGTCTTTCTGC

miR-766-5p	F TCGAGTACTTGAGATGGAGTTTT
	R GGCCGCGTTGCAGTGAGCCGAG

TRIM67	F TCCCAACTGTTTGCCACAGG
	R AGGTTAGAACGGAACGCCTC

U6	F CTCGCTTCGGCAGCACA
	R AACGCTTCACGAATTTGCGT

GAPDH	F AGCCTCAAGATCATCAGCAATG
	R TGTGGTCATGAGTCCTTCCACG

## Data Availability

The data used to support the findings of this study are available from the corresponding author upon request.
